The article "Monitoring of Sleep Breathing States Based on Audio Sensor Utilizing Mel-Scale Features in Home Healthcare" was published in 2023. Journal: J Healthc Eng.

# Monitoring of Sleep Breathing States Based on Audio Sensor Utilizing Mel-Scale Features in Home Healthcare

**DOI:** 10.1155/2023/6197564

**Published:** 2023-02-09

**Authors:** Yu Fang, Dongbo Liu, Zhongwei Jiang, Haibin Wang

**Affiliations:** ^1^School of Electrical Engineering and Electronic Information, Xihua University, Chengdu 610000, China; ^2^Graduate School of Science and Technology for Innovation, Yamaguchi University, Ube 755-0096, Japan

## Abstract

Sleep-related breathing disorders (SBDs) will lead to poor sleep quality and increase the risk of cardiovascular and cerebrovascular diseases which may cause death in serious cases. This paper aims to detect breathing states related to SBDs by breathing sound signals. A moment waveform analysis is applied to locate and segment the breathing cycles. As the core of our study, a set of useful features of breathing signal is proposed based on Mel frequency cepstrum analysis. Finally, the normal and abnormal sleep breathing states can be distinguished by the extracted Mel-scale indexes. Young healthy testers and patients who suffered from obstructive sleep apnea are tested utilizing the proposed method. The average accuracy for detecting abnormal breathing states can reach 93.1%. It will be helpful to prevent SBDs and improve the sleep quality of home healthcare.

## 1. Introduction

Healthcare-related issues have become the hot spots of society around the world. Among them, sleep quality plays an important role in health management. Poor sleep quality caused by sleep-related breathing disorders will impact peoples' daily life seriously. SBDs mainly include obstructive sleep apnea (OSA), central sleep apnea (CSA), and the mixed type. OSA which means the obstruction of the upper airway primarily due to the flabby tongue and uvula, is the most common SBD, CSA would cause sleep breathing apnea by the problem of the brain, and another type is the case mixed with the OSA and CSA [1]. The breathing abnormalities of SBDs are apnea, hypopnea, and snore. An apnea event lasts more than 10 seconds, and it can lead to a lower oxygen supply to the brain [2]. The ventilation of hypopnea will reduce to less than 50% ofnormal ventilation, and it will cause the value of oxygen levels to decline by more than 4% compared with the median. Snore is generated by a partial obstruction of the upper airway and is recognized as a vital sign of SBDs prevention [3]. The most harmful thing about these abnormal breathing states is the reduction of the oxygen supplement to the heart and brain. SBDs will lead to the complications of cardiovascular diseases and increase the risk of diabetes, cerebral stroke, and Alzheimer's disease [4, 5].

The article "Monitoring of Sleep Breathing States Based on Audio Sensor Utilizing Mel-Scale Features in Home Healthcare" was published in 2023. Journal: J Healthc Eng.

SBDs are not exclusive to the older as we thought, they will occur for different age groups and the morbidity is increasing in recent twenty years [6]. There is much evidence of the general population lacking awareness of SBDs, more than 20% of adults are suffering from SBDs with different levels, yet less than 25% of SBDs sufferers realized that they have been disturbed by the bad sleep health condition [1]. And the high cost of the existing clinical means keeps people from getting tests and treatment.

In the clinic, polysomnography (PSG) is the golden standard and the only way to provide the Apnea-Hypopnea Index (AHI) exactly for diagnosing SBDs. However, dozens of sensors used for PSG are not only costly but also complicated for common patients [7]. Hence, a smart and portable monitoring measure with the least sensors is imperative for home healthcare of SBDs.

The smart wearable with sensors is a new trend in the smart monitoring system of long-life diseases [8, 9], especially for the increasing demand for home healthcare. Researchers have applied different kinds of sensors, such as light sensors [10] and inertial sensors, to monitor the sleep condition by respiratory rate and breathing pattern analysis [11]. Researchers used the ultrasonic radar to normal and abnormal breathing activity [12] and used a thermal imaging camera to diagnose breathing disorders [13]. Researchers also used the sound sensors set near the nose and mouth to record the breathing sound signal for detecting apnea and hypopnea events by a set of pattern recognition rules [14]. Some researchers recorded tracheal signals from the throat to acquire the respiratory rate or set the sound sensor to the skin in a suprasternal notch to evaluate the breathing pattern in the high-frequency range [15, 16]. In previous studies, the sound sensors with smaller contact areas and easier operation are applied to record the breathing sound signal for sleep breathing monitoring [17]. As described above, these abnormal breathing states of SBDs will lead to decreasing ventilation while inspiration and expiration. The changes of ventilation can be reflected by different breathing states, such as snoring, apnea, hypopnea, and irregular breathing rate. Based on the production mechanism and physical significance of the abnormal breathing states, it is potential to detect the abnormality and health situation of sleep by breathing sound signals via a smart system with sound sensors.

In the research area of sleep monitoring based on breathing sound signals, many researchers focused on the respiratory rate detection based on the genetic algorithm [18], Hilbert transform [19], and neuro-fuzzy method [20] to analyze SBDs. In our previous study [21], a moment waveform analysis was proposed to segment the breathing cycles for respiratory rate detection. And snoring detection has been discussed to evaluate the level of SBDs [22]. And some researchers used the respiratory phase analysis to detect apnea [23]. Xie et al. proposed a deep learning method with a 2D spectrogram to detect snoring in various sleeping positions, based on constant *Q* transformation [24]. Shen et al. used CNN and LSTM to identify the snoring of OSAHS patients based on MFCC, LPCC, and LPMFCC and extracted the AHI index to evaluate the severity of OSAHS [25].

The article "Monitoring of Sleep Breathing States Based on Audio Sensor Utilizing Mel-Scale Features in Home Healthcare" was published in 2023. Journal: J Healthc Eng.

It can be found that the segmentation of breathing sound and the detection of breathing states are crucial for sleep monitoring and SBDs diagnosis. However, there are two problems. One problem is how to reduce the computational complexity of the analysis algorithms for the long-time data, that is, the real-time capability. Another one is how to guarantee the accuracy of the detection results. Most of the existed research always focused on a short period of the breathing signal, and the accuracy of the analysis results is not sufficient for healthcare. Our research aims to detect abnormal breathing states related to the SBDs such as apnea, hypopnea, and irregular breathing in a simple and fast way by a portable system.

This study keeps the ventilation of oxygen and carbon dioxide while sleep in mind and proposes a method to detect sleep breathing states based on Mel frequency cepstrum analysis by a portable acquisition system of breathing sound signal. In Section 2, the acquisition of breathing sound signal utilizing the sound sensor is introduced. The test condition and testers are also referred briefly. Then, the segmentation of breathing cycles is sketched in Section 3 as the preprocessing for the further analysis.  Section 4 describes the proposed detection method based on Mel frequency cepstrum analysis in detail, including the feature extraction and the identified rules of different sleep breathing states. Experiments and results can be found in Section 5. Finally, the discussion and conclusion are summarized in Sections 6 and 7, respectively.

## 2. Wearable Acquisition System with Sound Sensor

A wireless sound sensor and a commercial headset (Plantronics, M165) were applied to record sleep breathing data during the whole night. The M165 is very light and easily-operated. It is indeed a cheap and easy use for smart sleep healthcare in daily life. The acquired breathing data will be transmitted to a smartphone by Bluetooth and stored in mp3 format which is convenient for computerized analysis. The parameters of audio files can be set by an APP developed by our team. In this study, the sampling frequency is 44.1 kHz. The environment of data acquisition is shown in Figure 1. The headset is fixed to the nose by a strip of cosmetic tape. As we mainly focus on the changes in breathing airflow, the breathing sound signal from the nose and mouth can be recorded as long as the headset does not fall off and the tester is almost unaffected while sleeping whether at home or not.

The article "Monitoring of Sleep Breathing States Based on Audio Sensor Utilizing Mel-Scale Features in Home Healthcare" was published in 2023. Journal: J Healthc Eng.

At the beginning of preprocessing, the original sample frequency will be down-sampled to 11.025 kHz to reduce the computation amount. The real sleep breathing sound signal recorded by our system is shown in Figure 2.  Figure 2(a) is one-night sleep breathing sound data. The recording lasts about 5 hours, and the intensity of breathing changes greatly.  Figure 2(b) is a part of stable normal breathing sound data from the fifth hour and Figure 2(c) is a part of complex breathing sound data from the third hour. There are some obvious breathing pauses shown in Figure 2(c), and they are related to the obstruction of the airway. Hence, there is a high potential to identify different abnormal breathing states, such as apnea, hypopnea, unstable respiratory rate, and snore, from the breathing sound signal acquired via a portable and wireless sensor. Eight volunteers are selected as testers, including four in twenties, two in thirties, and two in Fifties. The study was approved by the ethics committee of Chengdu Region General Hospital (No. 2015 research 01). All testers' consent was obtained before participating in the study. The twenties and thirties were tested by Epworth sleepiness score (ESS), the scores were all less than 9, which was normal. The elder testers are diagnosed with moderate OSA and severe OSA by PSG with AHI=16 and 32, respectively. All the testers have monitored for the whole night lasting more than five hours. The breathing cycles of one-night data are counted, and the breathing states are manually labeled under the guidance of a professional physician for further analysis.

## 3. Segmentation of Sleep Breathing Signal Based on Characteristic Moment Waveform Analysis

To identify the breathing state accurately, the breathing cycle should be segmented for further analysis. A brief introduction of the segmentation method is presented in this section. The details can be found in our previous work [21].

The enhanced processing for amplitude contrast diminution has been performed first to reduce the effect of the weak breathing issues during the whole night's sleep.

The precondition assumes the noise part of the sleep breathing sound signal as a signal with zero-mean and unit variance. Suppose the sleep breathing sound signal is *r*(*t*), the random noise signal is *n*(*t*), and the real output signal is *y*(*t*)=*r*(*t*)+*n*(*t*), time characteristic waveform (TCW) of sleep breathing sound signal, denoted by *c*(*t*, *δ*), defined as the variance of the output *y*(*t*) can be given by the following equations:

(1) $$\begin{array}{c} c\left(t,\delta \right)=\int_{t-\delta }^{t+\delta }{\left(y\left(t\right)-\bar{y}\left(t\right)\right)}^{2}d\tau =\int_{t-\delta }^{t+\delta }y{\left(\tau \right)}^{2}d\tau -2\delta \bar{y}{\left(t\right)}^{2}\text{,} \end{array}$$

(2) $$\begin{array}{c} \bar{y}\left(t\right)=\frac{1}{2\delta }\int_{t-\delta }^{t+\delta }y\left(\tau \right)d\tau \text{.} \end{array}$$

Then, the characteristic moment waveform (CMW) is calculated by the thought of image shape identification in image processing with another time scale *l*, which is represented by *I*(*t*, *δ*, *l*). It is calculated according to the following equation:

(3) $$\begin{array}{c} I\left(t,\delta ,l\right)=\int_{t-l}^{t+l}{\left(\tau -t\right)}^{2}c\left(\tau ,\delta \right)d\tau \text{.} \end{array}$$

For a discrete signal with length *N*, the computations of TCW and CMW only need 8 *N* and 15 *N* additions and multiplications, respectively. The algorithm can process the whole night data fast, and it will be helpful for real-time motoring.

The article "Monitoring of Sleep Breathing States Based on Audio Sensor Utilizing Mel-Scale Features in Home Healthcare" was published in 2023. Journal: J Healthc Eng.

According to our experimental statistic, the scale *l* is usually set to (1.5, 3), about half of the sleep breathing cycle. The time scale *δ* is set as 0.1, about 1/10 of the phase duration. After choosing the suitable time scales, TCW and CMW can be extracted by equations (1) to (3). *C*_min_ of CMW is the local minimum point sequence which would be calculated first. Then, the local maximum points sequence *T*_max of TCW can be found by a computation window with *C*_min_ as the central points. The local maximum point sequence of CMW can be obtained as the cycle segmentation points and adjusted according to *T*_max. Finally, the incorrectly segmented breathing pauses will be combined utilizing a threshold value by the average amplitude of the test data.

The breathing cycle segmentation result of partial normal breathing signal is shown in Figure 3.

## 4. Detection of Breathing States via Mel Frequency Cepstrum Analysis

During the whole night's sleep, the sleep breathing state changes greatly. Besides the apnea, there are the hypopnea events, snore events, and others as shown in Figure 4. In Figure 4, two types of irregular breathing events are found and shown by blue and orange boxes. They are all related to the obstruction of the upper airway. The breathing parts marked by blue boxes display the changed respiratory rate. By hearing, they mix with noise caused by the movements of the nose and mouth. It is easy to find that the breathing parts of orange boxes have higher amplitude with the extended or merged inspiration/expiration. And they sound similar to labored breathing and can be classified as a kind of snore.

The article "Monitoring of Sleep Breathing States Based on Audio Sensor Utilizing Mel-Scale Features in Home Healthcare" was published in 2023. Journal: J Healthc Eng.

Differing from the apnea with a clear definition in the time domain, other complex breathing states cannot be detected in the time domain. According to the previous research, the distribution of frequency energy would be very different between the normal and abnormal breathing states. From the time-frequency representation, the breathing case with apnea has much more energies below 500 Hz and above 3500 Hz compared with the normal case. It provides a probable way to distinguish the different breathing states in the frequency domain.

### 4.1. The Conventional MFCCs Analysis

Psychophysical studies have shown that human perception of the frequency content of sounds does not follow a linear scale. The Mel frequency cepstrum coefficients (MFCCs) were proposed as it is very similar to perceptual linear predictive analysis of sound [26]. MFCCs were derived from the short time spectrum of a signal and were widely used both for speech and speaker recognition [27, 28]. MFCCs have already been applied to extract features of respiratory sound in combination with learning machines to recognize the wheeze for respiratory disorders [29, 30].

First of all, framing and windowing are applied for the conventional MFCC algorithm. Then, fast Fourier transform (FFT) is used to transform the signal of each frame from the time domain to the frequency domain. Then, the energy spectrum is calculated. Next, the energy signal is filtered by the Mel-scale filter bank and processed in the logarithm orderly. At last, discrete cosine transform would transform the signal into the time domain and extract a series of coefficients.

As the core of MFCCs, the relationship between Mel frequency and real frequency is defined as follows:

(4) $$\begin{array}{c} Mel\left(f\right)=\frac{1000*\;\mathrm{lg}\;\left(1+\left(f/700\right)\right)}{\mathrm{lg}\;\left(1+\left(1000/700\right)\right)}\text{,} \end{array}$$

where *f* is the real frequency and Mel(*f*) is the Mel-scale frequency. As the human perception of the frequency content is almost linear below 1 kHz and nonlinear over 1 kHz, 1000 is a key parameter to determine the relationship of *f* and Mel(*f*) simulating the character of the human ear. 700 is the parameter that affects the relationship's changing trend between *f* and Mel(*f*).

For the frequencies under 1000 Hz, the Mel scale can be approximated to a linear scale. Mel frequency can represent the details of the low-frequency range more accurately than the high-frequency range. Hence, it can capture formants that lie in the low-frequency range.

The article "Monitoring of Sleep Breathing States Based on Audio Sensor Utilizing Mel-Scale Features in Home Healthcare" was published in 2023. Journal: J Healthc Eng.

The Mel filter bank is designed based on Mel-scale frequency. The Mel-scale frequency distributes uniformly-spaced in Mel scale, simulating the critical frequency bands of the human ear. The center of each triangle window is the starting of the next one.

The logarithm is used to compress the components above 1000 Hz. And it can translate the multiplicative components into the additive ones and reduce the computation complexity [26]. A logarithm can provide the frequency energy distribution of a one-time point in the form of addition. Finally, the Mel frequency cepstrum coefficients will be extracted by discrete cosine transform.

Our purpose is to find the relationship between the frequency energy distribution and the monitoring time. The results of the processing after the logarithm should be paid attention to in this study.

### 4.2. Analysis of Breathing Sound Signal Based on Mel Frequency Cepstrum Analysis

Here, we proposed a method of parameters extraction to detect different breathing states, and the flowchart is displayed in Figure 5.

As shown in Figure 5, window screening is the first step and the length of the rectangle window is set as 1024 sample points, about 100 ms according to the sampling frequency. The window moves foreword by overlapping the half of itself to keep enough details of the observation. Then, the frequency energy distribution of the breathing sound signal would be calculated by power spectrum density (PSD) in the second step. The PSD estimation is an important part of modern signal processing and reflects the energy distribution of the frequency component of the signal. The autoregressive (AR) method is the most frequently used parametric method because the estimation of AR parameters can be performed easily by solving the linear question. Here, Yule–Walker's method is used to make the power spectrum density instead of the energy of the FFT result. The order of an autoregressive prediction model for the signal is set as 32 [31].

In the third step, the energy of the signal is filtered by the Mel frequency filter banks including 20 triangle filters. The triangle filter bank is selected by default in speech processing shown in Figure 6, which simulates the auditory characteristics of the human ear. The mathematical expression of the triangular window is simple, reducing the amount of computation.

And the 20-dimension Mel-scale features are extracted after the logarithm operation in the fourth step. The horizontal of the feature matrix represents frames of observation time. The vertical of the matrix represents the Mel-scale filters of the filter bank.

The article "Monitoring of Sleep Breathing States Based on Audio Sensor Utilizing Mel-Scale Features in Home Healthcare" was published in 2023. Journal: J Healthc Eng.

To stand out the frequency energy distribution of each frame, a new feature set has been proposed in the fifth step, the core of our proposed method. The procedure of the proposed method to extract the effective features is described in detail. The sketch map of extraction for one breathing cycle can be found in Figure 7 to illustrate the algorithm.

- Extract the Mel-scale features of one segmented breathing cycle according to the first four steps of the flowchart in Figure 5.
- The Mel-scale features *f*_*i*,*j*_ can be displayed by the stretch map shown in Figure 7(b). *i* is the label of the triangle filters of the Mel frequency filter bank in the frequency domain, from 1 to 20. *j* is the number of frames in the time domain, from 1 to *N*. *N* is the total number of frames of each breathing cycle.
- Find the maximum point of each column of *f*_*i*,*j*_, denoted by *A*_*i*,*j*_.
- *i* is corresponding to the label of the Mel-scale filter and represents a fixed Mel-scale frequency range. We proposed it as Mel-scale label (MsL) as shown in Figure 7(c). The *X*-axis is the frame number, and *Y*-axis is the Msl. MsL can be explained by the main part of frequency energy distributing in one observed duration in the time domain.
- Compute the present times of each MsL to represent the distribution of frequency energy in each cycle, marked as *N*_MsL_ which is shown in the bar chart of Figure 7(d). MsL and *N*_MsL_ are proposed to detect the abnormal breathing sound signal. For the normal breathing cycle shown in Figure 7(a), it is found that the label number *i* of MsL is from 4 to 14 in the duration of inspiration and expiration compared with the breathing stopping intervals as shown in Figure 7(c). So, the frequency energy of this breathing cycle is mainly filtered by the No. 4 to No. 14 Mel-scale filter as same as the results of *N*_MsL_ shown in Figure 7(d).

After all the five steps, we can use MsL and *N*_MsL_ to analyze the components of the breathing sound signal and to detect the abnormal breathing states finally. The results of detecting abnormal breathing states will be demonstrated in the next section.

## 5. Experiment

### 5.1. Analysis of Breathing Sound Signal by the Proposed Identification Method

The label of Mel-scale features, MsL, and the corresponding *N*_MsL_ in each segmented breathing cycle during one-night monitoring can be extracted. The energy of distribution in a fixed frequency range is useful to present the features of different breathing states. We mainly separate snoring, normal breathing, and abnormal breathing components of the breathing signal.

The article "Monitoring of Sleep Breathing States Based on Audio Sensor Utilizing Mel-Scale Features in Home Healthcare" was published in 2023. Journal: J Healthc Eng.

It is found that the MsL in the low-frequency range can represent the snore component. The normal breathing component is usually represented by MsL in the middle-frequency range. The abnormal breathing components including apnea, hypopnea, and irregular breathing rate can be expressed by MsL in the high-frequency range. Checking results manually by ear and eye is the reference under the guidance of a professional doctor.

So, three MsL sets are proposed, i.e., low-frequency label set, middle-frequency label set, and high-frequency label set and marked as FL, FM, and FH, respectively, in Figure 8.

For different individuals, there would be a little difference when we partition these three MsL sets. Based on the experimental attempts, the common part of each MsL set is selected for the further analysis, that is, MsL_2_ for the snore detection, MsL_4_ to MsL_7_ for the normal breathing state detection, and MsL_15_ to MsL_17_ for the abnormal breathing state detection. To detect different breathing components in each breathing cycle, threshold values are applied and displayed by red lines in Figure 8. As the time duration of inspiration and expiration lasts about 2.5 seconds in one breathing cycle according to our experimental dataset, the total *N*_MsL_ equals the total number of frames, about 50 times. Hence, according to the experiment results and observation, the threshold values for FM and FH are set by 40% of the total *N*_MsL_ of each MsL, about 20 times. And the threshold value of FL is set by 20% of the total number *C*_*L*_*i*__ of each MsL, about 10 times.

If *N*_MsL_ is larger than the red threshold line, the corresponding cycle can be symbolized by 1, the opposite is 0. It is obvious that the breathing cycles with abnormal component always accompany the snoring component. The abnormal component and normal component do not exist at the same time in the usual case from Figure 8. So, it is the potential to detect different kinds of breathing states based on these three MsL sets.

If there is ‘1' of FH, the breathing state can be detected as abnormal. If there is ‘0' of FH, combined with the detection results of FM, heavy breathing can be identified from the normal states which can be checked by the ear.

The snore can be divided into the normal type and the abnormal type. Normal snore is related to simple snoring, and abnormal snore is related to SBDs. However, they all should be concerned. So, the snore is detected separately from other abnormal breathing states and listed for a useful index. If there is ‘1' in FL, the breathing cycle is identified as breathing with snore.

The study focuses on the ratio of abnormal breathing states during the monitoring for sleep healthcare management in the early stage. Obviously, the subclassifying of breathing types is a rough judgment now and it will be applied to a deeper discussion of accurate analysis for SBDs in the future work.

The article "Monitoring of Sleep Breathing States Based on Audio Sensor Utilizing Mel-Scale Features in Home Healthcare" was published in 2023. Journal: J Healthc Eng.

### 5.2. Application for the Sleep Breathing States Detection

The identified results by MsL sets for an OSA tester (AHI=16) are shown in Figure 9.  Figure 9(a) displays the detection results of normal/abnormal sleep state. The abnormal sleep breathing cycle is denoted by ‘1' and the normal sleep breathing is ‘0' based on the identification rules introduced in the last subsection. It is easy to compute the time duration of normal and abnormal breathing state lasting during the whole night. In this case, the normal breathing lasts 2.8 hours, and the abnormal breathing lasts 2.2 hours.  Figure 9(b) displays the detection result of snoring. The breathing cycle with snore is marked as ‘1,' and the snore lasts 1.8 hours of the whole night totally.

The time duration of breathing stop from the audio waveforms can distinguish the apnea and typical hypopnea from normal breathing states. For apnea, the breathing stop is larger than 10 s. As the ventilation of hypopnea will reduce to less than 50% of the normal ventilation, the breathing stop of the typical hypopnea is calculated from 6 s to 10 s according to the clinical definition of apnea and hypopnea [2]. Irregular breathing rate can be picked up by comparing with the normal parts.

From the original breathing waveforms of *A*1 to *A*3 shown in Figure 10, two parts of the breathing signal in each section are shown orderly. It can be found that there is obvious apnea (such as *A*1-1, *A*3-1, and *A*3-2), hypopnea (such as *A*1-2), irregular breathing (such as *A*1-1, *A*2-1, and *A*2-2), and breathing with noise caused by the body movement (such as *A*2-1) from the waveforms in time domain clearly. Sections *A*1 to *A*3 belong to the abnormal breathing states with snore.

From the original breathing waveforms of *N*1 and *N*2 shown in Figure 11, these two sections are normal stable breathing, and breathing of *N*2 is snoring. The red line in Figure 10 is the envelope of the spectrum, and it is easy to find that there is a large energy in the middle-frequency range (500–1500 Hz), representing the normal breathing component for both *N*1 and *N*2. The amplitude of *N*2 is higher than *N*1. And the higher ratio of frequency energy distributes below 500 Hz is the main feature of snore shown in section *N*2.

Applying the proposed method based on Mel-scale features, the monitoring results of all the testers are listed in Table 1. We can find the total time of the whole night monitoring and the time durations of different breathing states. To evaluate the sleep quality, the ratio of the normal breathing during the night is computed by the following equation:

(5) $$\begin{array}{c} R_{Sleep}=\frac{T_{Normal}}{T_{Monitoring}}\text{,} \end{array}$$

where *R*_Sleep_ is used to test the quality of sleep by the detection of normal breathing state, *T*_Normal_ is the total time duration of normal breathing state lasting, and *T*_Monitoring_ is the total time duration of the sleep monitoring. It will be a meaningful index to know and manage sleep health in one's daily life.

The article "Monitoring of Sleep Breathing States Based on Audio Sensor Utilizing Mel-Scale Features in Home Healthcare" was published in 2023. Journal: J Healthc Eng.

According to the detected results of breathing states, the ratio of normal breathing states is over 70% for testers no. 1, 2, 3, and 5 which is higher than the OSA testers no. 7 and 8, which were diagnosed by PSG. Testers No. 4 and 6 have lower ratios of normal breathing state and there are indeed a lot of apnea and hypopnea events during the monitoring procedure by checking up on the original breathing signal. Testers no. 4 and 6 were diagnosed as severe rhinitis by the doctor during the experimental period. Actually, after the relief from rhinitis symptoms, the results of monitoring are within the normal range. The extreme cases of young testers can also show the efficiency of the proposed method.

Moreover, it is found that the testers with a low ratio of normal breathing state always snore with a longer time duration. Hence, snore is really an important sign related to the analysis and prevention of sleep breathing-related disorders.

The accuracy of detecting normal and abnormal breathing states can be given based on the prepared manual labels in our experiment, and the accuracy of our proposed method of the testers can reach 95.2% shown in Table 1, and the average value is 93.1%.

## 6. Discussion

In the studies of breath state detection by breath sound signal, some researchers used the measurement of energy to detect apnea events during the breath and breath hold [23]. From [24] in Table 2, it can be seen that the MFCC feature parameters are the most effective in classifying snores among the three features used. Using MFCC combined with the LSTM method can achieve 87% accuracy. At the same time, the AHI index was also estimated. Although there is a particular gap with the AHI value detected by PSG, it can be used as an auxiliary reference in the classification of OSAHS. It can also be found that the average accuracy of snoring recognition of OSA patients and normal people is 95.3% by combining deep learning and two-dimensional spectral features in [25]. Literature [23] used spectral energy and VAD criterion threshold for apnea detection for simulated apnea signals and achieved an accuracy of 97%. Still, it is not applied to the actual breathing signals of OSA patients, nor does it mention hypopnea detection.

The article "Monitoring of Sleep Breathing States Based on Audio Sensor Utilizing Mel-Scale Features in Home Healthcare" was published in 2023. Journal: J Healthc Eng.

The method in this paper does not use classical machine learning and deep learning methods, so the amount of calculation is small. Moreover, the threshold displays the fact between the characteristic parameters and the breathing signal. At the same time, the normal and abnormal breathing and snoring sounds are distinguished. The accuracy rate of 93.1% can be achieved by judging normal and abnormal breathing. The judgment of abnormal breathing includes apnea, hypopnea, and other respiratory disturbance events. However, due to the small amount of breathing data and individual differences among testers, there is a state of misjudging normal breathing as snoring in snoring detection. It is necessary to refine the types of abnormal breathing and accurately find them for the intervention in continuous work.

Some researchers combined a sound sensor, accelerometer, and pulse oximeter to get AHI index for SBDs [16]. Moreover, the degree of blood oxygen saturation (SpO2) acquired by the pulse oximeter is a vital index for the respiratory system in the clinic. The SpO2 will decrease when there is an obstruction in the upper airway; that is, apnea, hypopnea, and irregular breathing will accompany the lower value of SpO2.

Hence, SpO2 has been monitored for the testers as well and the abnormal breathing states can be evaluated by subtracting a fixed value from the medium value of SpO2. In our experiment, it is easy to find that the results of SpO2 are included in the scope of the proposed detection. The comparison results with SpO2 are given in Figure 12. The red line represents the median value of the tester's SpO2. It can be seen that the period when SpO2 has a significant decrease compared to the median value is detected as an abnormal breathing state which matches the detection results.

However, the abnormalities caused by the light obstruction of the airway can be pointed out by the proposed detection, which is not clearly defined. It may be related to the threshold values set by our proposed detection. More types of abnormal breathing states will be discussed deeply in future work. And because the tapes may become loose and the microphone's location may change occasionally, the acquisition system should be developed. And the classification and identification of breathing states are further refined. The analysis of the hypopnea state is limited by the small amount of experimental data and cannot be further refined and analyzed.

In other words, the tester dataset should be enlarged and the types of abnormal breathing states should be discussed in detail. We will optimize the ranges of MsL sets to analyze the components of breathing sound signal, such as dividing different frequency ranges to show more precise results. The relationship between our definitions of abnormal breathing and the pathological characteristics of SBDs will be discussed deeply in further study.

The article "Monitoring of Sleep Breathing States Based on Audio Sensor Utilizing Mel-Scale Features in Home Healthcare" was published in 2023. Journal: J Healthc Eng.

## 7. Conclusion

In this study, the sound sensor and microphone in a headset with Bluetooth were utilized to record and transmit the breathing sound signal during the whole night. The portable and wireless acquisition system proposed in this paper has less impact on sleep quality and can be operated simply anywhere. And the MFCCs are introduced from speech signal processing to the processing of breathing signal for sleep monitoring in-home healthcare. The MsL representing the main distribution of frequency energy in each frame is proposed to detect the different sleep breathing states. In addition, the data acquisition operation is simple, the cost of detection is low, and the accuracy can satisfy individual monitoring needs. Recognition of respiratory status and detection of abnormal breathing can be popularized in daily monitoring. It can also be used as an aid for clinical diagnosis based on a more detailed analysis of the results. The study is limited by the small amount of experimental data, so the classification and identification of breathing need to be further improved, and the adaptability and accuracy of the algorithm need to be further enhanced. Although it has particular reference significance for the long-term sleep monitoring of individuals, the algorithm is still unstable in monitoring different people.

The core of the Mel frequency analysis is to reflect the relationship between the monitoring time and the frequency energy simulating the acoustic character of the human ear. For each frame in the time domain, the MsL is extracted by finding the maximum value of the frequency energy in each Mel scale. Then, the present times of each MsL are computed to show the frequency energy distribution of each segmented breathing cycle. Three MsL sets are determined corresponding to the normal breathing component, abnormal breathing component, and snore component, denoted by FM, FH, and FL. Finally, with the suitable threshold values and comprehensive evaluation rules, the normal breathing state, abnormal state, and snore state can be detected successfully. The types of sleep breathing states should be discussed deeply and classified accurately for examination and analysis of SBDs. And for different individuals, long-time monitoring and big data analysis are necessary to acquire more precise monitoring results for the prevention and treatment of SBDs in the future.

The article "Monitoring of Sleep Breathing States Based on Audio Sensor Utilizing Mel-Scale Features in Home Healthcare" was published in 2023. Journal: J Healthc Eng.

## Figures and Tables

**Figure 1:** The wearable acquisition system via a wireless sensor.

**Figure 2:** The original waveforms acquired by the portable system. (a) The sleep breathing sound signal of one-night test; (b) the part of normal breathing signal from recording 2(a); and (c) the part of abnormal breathing signal from recording 2(a).

**Figure 3:** Segmentation result by CMW.

**Figure 4:** Three parts of abnormal sleep breathing sound data.

**Figure 5:** The flowchart of the modified Mel frequency cepstrum analysis.

**Figure 6:** Schematic diagram of the triangular filterbank.

**Figure 7:** Extraction of Mel-scale indexes for a breathing cycle. (a) The waveform of a breathing cycle; (b) the sketch map of Mel-scale features; (c) the 1st index, MsL; and (d) the 2nd index, *N*_MsL_.

**Figure 8:** *N*_MsL_ of FL, FM, and FH is used to detect breathing components.

**Figure 9:** Monitoring results by MsL sets for an OSA tester. (a) Detection of normal and abnormal breathing states. (b) Detection of snoring state.

**Figure 10:** Validation of the abnormal breathing state detection by the proposed method.

**Figure 11:** Validation of the normal breathing state detection by the proposed method.

**Figure 12:** Comparison detection results with SpO2.

**Table 1:** Detection results of sleep breathing states of testes.

Tester no	Years	Time (hour)	Normal (hour)	Abnormal (hour)	Snoring (hour)	Accuracy of *S*/*N*(%)	Normal ratio (%)	Accuracy of *A*/*N*(%)
1	20	7.7	6	1.7	0.5	93.5	77.9	93.2
2	21	7.5	5.6	1.9	0.3	96.0	74.7	94.4
3	21	6.8	4.9	1.9	0.1	98.5	72.1	91.9
4	20	6	2.4	3.6	2.2	96.4	40	90.2
5	31	7.5	5.5	2	1	90.8	73.3	94.9
6	34	8	4.2	3.8	3.2	97.6	52.5	92.2
7	58	5	2.8	2.2	1.8	97.5	56	95.2
8	60	6.8	2.3	4.5	3.8	98.2	33.8	92.7

**Table 2:** Summary of previous studies on breathing states detection by acoustic signal.

Authors	Method	Features	Dataset	Snore detection results	Abnormal detection results
[23]	Voice activity detection algorithm	FFT	50 normal people breath 20 cycles and hold their breath to make the apnea	Not mentioned	Apnea detection accuracy more than 97%
[24]	CNN + RNN	CQT spectrogram	Part of full night recordings from 38 subjects	Accuracy: 95.3%	Not mentioned
[25]	CNN + LSTM	MFCC, LPCC and LPMFCC	Whole night recoding from 32 volunteers	Accuracy: 87%	Calculate AHI values
This study	Threshold values for individuals	Mel-scale-based features	Full nights recoding from 8 testers	Accuracy: 96.1%	Accuracy: 93.1%

## Data Availability

The data used to support the findings of this study are available from the corresponding author upon request.
